This article has been retracted.

# LINC00346 Acts as a Competing Endogenous RNA Regulating Development of Hepatocellular Carcinoma via Modulating CDK1/CCNB1 Axis

**DOI:** 10.3389/fbioe.2020.00054

**Published:** 2020-02-18

**Authors:** Jinglan Jin, Hongqin Xu, Wanyu Li, Xiaotong Xu, Huan Liu, Feng Wei

**Affiliations:** ^1^Department of Hepatology, The First Hospital of Jilin University, Changchun, China; ^2^Department of Hepatobiliary and Pancreatic Surgery, The First Hospital of Jilin University, Changchun, China

**Keywords:** LINC00346, miR-1991-3p, CDK1, CCNB1, p53 signaling pathway, hepatocellular carcinoma

## Abstract

Hepatocellular carcinoma (HCC) is one of the important types of liver cancer. LncRNA is an important regulatory factor that regulates many biological processes such as tumor cells during tumorigenesis and metastasis. LINC00346 has been associated with various types of liver cancer, but its role and regulatory mechanism in HCC remain unclear. In our study, we found the LINC00356-miR-199a-3p-CDK1/CCNB1 axis through bioinformatics analysis. The expressions of LINC00356, miR-199a-3p, CDK1, and CCNB1 in HCC and normal hepatocytes were determined by qRT-PCR and WB. The results showed that LINC00356, CDK1 and CCNB1 were highly expressed in HCC, while miR-199a-3p was lowly expressed. Dual luciferase reporter gene assay, RIP and RNA-pull down assays demonstrated the targeted binding relationship of LINC00346-miR-199a-3p-CDK1/CCNB1. Overexpressing LINC00460 and silencing miR-199a-3p promoted cell invasion, inhibited apoptosis of HCC, and arrested the cell cycle in S phase while opposite results were obtained when silencing LINC00346, CDK1, and CCNB1. LINC00346 indirectly affects liver cancer by promoting the expression of CDK1/CCNB1 through competitive adsorption of miR-199a-3p. In addition, the study also demonstrated that overexpression of LINC00346 indirectly inhibited the expression of p53 and p21 proteins by promoting CDK1/CCNB1 expressions, thereby blocking the p53 signaling pathway. These results proved that LINC00346 could regulate the expression of CDK1/CCNB1 through the competitive adsorption of miR-199a-3p, thereby affecting the p53 signaling pathway and finally regulating the apoptosis, invasion and cell cycle of HCC cells. In conclusion, LINC00346 can be used as a tumor promoter and potential therapeutic target for HCC metastasis and prognosis.

## Introduction

Primary liver cancer is one of the second leading causes of death worldwide, and hepatocellular carcinoma (HCC) is one of the major types of it (Sia et al., 2017). In recent years, incidence rates continue to increase rapidly for liver cancer, by about 3% per year in women and 4% per year in men (Siegel et al., 2017). Although the treatment of HCC has improved significantly in recent decades, including surgical resection, liver transplantation, radiotherapy and chemotherapy, the overall 5-year survival rate is not improved (Ulahannan et al., 2014). Over the years, the occurrence of liver cancer is considered to be a complex multi-step process involving multiple molecules and multiple signaling pathways (Setshedi et al., 2018). A better understanding of the occurrence and development of HCC will help to further improve treatment strategies. Therefore, it is of great significance to explore the mechanism of the occurrence and development of HCC, determine the effective therapeutic targets of HCC, and find a new way for HCC treatment.

Recently, increasing evidence confirms that long non-coding RNAs (lncRNAs) and microRNAs (miRNAs) have been identified as important regulators in a variety of cancers including HCC (Bartel, 2004; Li and Chang, 2014; Wang et al., 2017). Abnormal expression of lncRNA plays a key role in cancer progression and carcinogenesis through a variety of mechanisms (Chen et al., 2016). LINC00346 is located on chromosome 13q34, with a total length of 6322bp, and is up-regulated and has oncogenic effects in non-small cell lung cancer and bladder cancer (Ye et al., 2017; Zhang B. et al., 2018). Overexpression of LINC00346 was positively correlated with poor prognosis of pancreatic cancer (Brown et al., 2018). Zhang et al. (2015) have found that the up-regulated expression of LINC00346 in HCC is significantly negatively correlated with the survival of HCC patients. These results indicate that LINC00346 plays a significant oncogenic role in a variety of cancers, but the specific biological function and mechanism of LINC00346 in HCC have not been studied.

Cyclin-dependent kinase (CDK) is an important cell cycle-regulating protein, belonging to the serine/threonine kinase family, which includes catalytic kinase subunits and cell cycle protein conjugates. Only CDK1 in the CDK family can promote cell cycle independently (Santamaría et al., 2007; Malumbres and Barbacid, 2009). CDK1 has been reported to be highly expressed in human colorectal cancer (Sung et al., 2014), prostate cancer (Willder et al., 2013). Therefore, CDK1 is closely related to cancer progression. In the study of the specific role of CDK1 in cancer. Danhier et al. (2010) have reported that CDK1/CyclinB1 inhibitor JNJ-7706621 and aurora kinase combined with paclitaxel can effectively treat transplantable liver cancer and inhibit tumor growth. In addition, studies have shown that CDK1 and CCNB1 have inhibitory effects on p53 signaling pathway as regulatory factors in HCC (Qin et al., 2019). Cell cyclin B1 (CCNB1) is an important cell cycle protein whose abnormal expression plays an important role in regulating cell cycle (Jin et al., 1998). Recent studies have demonstrated that CCNB1 is highly expressed in various human cancers, including breast cancer (Niméus-Malmström et al., 2010), cervical cancer (Kreis et al., 2010) and lung cancer (Yoshida et al., 2004). Moreover, Porter et al. (2003) found that inhibition of CCNB1 nuclear export and CCNB1 accumulation in the nucleus induced apoptosis. CCNB1 has also been proved to significantly correlate with overall survival of HBV-related HCC recurrence. These results indicate that CDK1/CCNB1 are significantly positively correlated with the development of various cancers including HCC, but the specific role of these two genes in HCC has not been investigated.

In this study, we found that LINC00346 was highly expressed in HCC cells, and it regulated the expressions of CDK1/CCNB1 through competitive adsorption of miR-199-3p as a ceRNA, thereby promoting the proliferation and metastasis of HCC cells. LINC00346 also regulated the p53 signaling pathway by regulating the miR-199-3p/CDK1/CCNB1 signaling axis. These results demonstrated that LINC00346 played a significant oncogenic role in the development of HCC and LINC00346 can be used as a prognostic target and potential biomarker in the diagnosis and prognosis of HCC.

## Materials and Methods

### Bioinformatics Analysis

Hepatocellular carcinoma expression datasets GSE62232 (including 10 normal samples and 81 HCC samples) and GSE74618 (including 10 normal samples and 218 HCC samples) were obtained through GEO database^1^. Normal samples were set as control, and “limma” package was used for differential analysis with the threshold of |logFC| > 2 and *P*-value < 0.05. KEGG pathway enrichment analysis of the differential genes was conducted by “clusterprofiler” package, and the pathview diagram was plotted by “pathview” package. Gene interaction analysis was conducted through STRING database^2^, and gene interaction network map was drawn by cytocape v3.7.1. The expression levels of CDK1 and CCNB1 in TCGA^3^ database were retrieved through GEPIA database^4^. The upstream regulatory miRNAs of CDK1 and CCNB1 were predicted and the binding site information of miRNA-mRNA was obtained by TargetScan database^5^. The upstream lncRNAs of miR-199a-3p were predicted by RAID database^6^, and lncRNA-miRNA binding site information was obtained through RNA22 database^7^.

### Cell Lines and Transfection

Human normal liver cells L-02 (BNCC351907), HCC cell lines HepG2 (BNCC338070), Huh-7 (BNCC337690), Hep3b (BNCC337952), and SMMC-7721 (BNCC352197) were all purchased from BeNa Culture Collection. All cell lines were incubated with 90% Dulbecco’s Modified Eagle Medium (DMEM)-H containing 10% fetal bovine serum (FBS, Gibco, Grand Island, NY) and maintained in an incubator with 5% CO_2_ at 37°C.

LINC00346, oe-LINC00346, CDK1 and CCNB1 siRNA, miR-199a-3p inhibitors, miR-199a-3p mimic or corresponding controls were obtained from GENECHEM (Shanghai, China) and transfected into cells in 6-well plates by Lipofectamine 3000 (Invitrogen, United States) according to the manufacturer’s instructions. In addition, PFT β [Pifithrin-β, p53 protein inhibitor, HY-16702, MedChemExpress (Da Pozzo et al., 2014)] was added to the culture medium at 10 μM per well plate. All cells were transfected for 48 h and collected for subsequent experiments.

### qRT-PCR

Total RNA from transfected cells was extracted by TriZol reagent (Qiagen) according to the instructions. Complementary DNA (cDNA) synthesis and quantitative polymerase chain reaction (qPCR) procedures were performed for mRNA and lncRNA using PrimeScript RT Master Mix and TB Green Premix Ex Taq II (TaKaRa, Dalian, China). RNA of miRNA was isolated using the miRNeasy Mini Kit (Qiagen, Shenzhen, China). Mir-x miRNA first strand synthesis kit and Mir-x miRNA quantitative real-time polymerase chain reaction (qRT-PCR) SYBR kit (TaKaRa) were used for reverse transcription and qPCR. The primers were listed in Table 1. U6 snRNA was used as an internal reference for miR-199a-3p, and GAPDH was the internal reference of LINC00346, CDK1 and CCNB1. The data were analyzed by 2^–Δ^ ^Δ^ ^*Ct*^ method.

**TABLE 1:** Primer sequences.

Genes	Primer sequences
LINC00346	F: 5′-TCTCACCAGCATTTGACGCT-3′
	R: 5′-ACGTGCGCAAGTAAGTCTCA-3′
CDK1	F:5′-AAACTACAGGTCAAGTGGTAGCC-3′
	R:5′-TCCTGCATAAGCACATCCTGA-3′
CCNB1	F:5′-GACCTGTGTCAGGCTTTCTCTG-3′
	R:5′-GGTATTTTGGTCTGACTGCTTGC-3′
GAPDH	F:5′-CAGGAGGCATTGCTGATGAT-3′
	R:5′-GAAGGCTGGGGCTCATTT-3′
miR-199a-3p	F:5′-CTCACAGTAGTCTGCACA-3′
	R:5′-GACTGTTCCTCTCTTCCTC-3′
U6	F:5′-CTCGCTTCGGCAGCACA-3′
	R:5′-AACGCTTCACGAATTTGCGT-3′

### Western Blot (WB)

Total protein was extracted from transfected cells by RIPA lysis buffer (Beyotime, Shanghai, China). The purity of the protein in the whole extract was determined by bicinchoninic acid (BCA) protein assay kit (Pierce, Appleton, WI). The proteins were separated by SDS-PAGE and transferred to PVDF membrane (Millipore). After incubation with bovine serum albumin (BSA) in Tris-HCl buffered saline containing 0.1% TBST, the membrane was added with corresponding primary antibodies CDK1 (ab32094, 1:2000, Abcam, Cambridge, MA), CCNB1 (ab32053, 1:50000, Abcam, Cambridge, MA), p53 (ab32389, 1:1000, Abcam, Cambridge, MA), p21 (ab109520, 1:1000, Abcam, Cambridge, MA), and GAPDH (ab181602, 1: 10, 000, Abcam, Cambridge, MA). Second antibody Goat anti-rabbit IgG H&L (horseradish peroxidase, HRP) (ab6721, 1:2000, Abcam, Cambridge, MA, United States) was then used to incubate the membrane. The positive bands were detected by Immobilon Western Chemiluminescent HRP Substrate (Millipore) and the strength of the target strip was quantified by Image Lab Software (Bio-Rad).

### Flow Cytometry (FCM)

Apoptosis assay: transfected cells for 48 h were collected and the apoptosis rate was measured by Annexin V-FITC/PI apoptosis assay kit (Beijing Biosea Biotechnology, Beijing, China). In brief, the cells were stained with 10 μL Annexin V-FITC and 5 μL propidium iodide (PI). After incubation in darkness at room temperature for 30 min, the samples were analyzed by FCM (Beckman Coulter, Fullerton, CA, United States). Annexin V-PE (+)/PI (-) represents apoptotic cells, while Annexin V-PE (+)/PI (+) represents early apoptotic or dead cells.

Cell cycle determination: after transfection for 48 h, cells were harvested and stained with PI using the CycleTest Plus DNA Reagent kit (BD) in accordance with the manufacturer’s guidelines. Finally, the percentage of cells in G0/G1, S and G2/M phases was counted.

### Transwell

Invasion measurement was performed using Transwell Chambers consisting of an 8 μm membrane filter (Corning Incorporated, Corning, NY, United States) coated with Matrigel (BD Biosciences, San Jose, CA, United States). Cells were trypsinized and suspended in serum-free medium. Next, 2 × 10 (Setshedi et al., 2018) cells were plated in the upper chamber, and the lower chamber was filled with a medium containing 10% FBS. After incubation for 36 h, the cells in the lower chamber were fixed with 4% paraformaldehyde and stained with crystal violet. Five fields were randomly selected and cells were counted under a microscope.

### RIP Assay

The EZ-magna RIP kit (Millipore, United States) was applied to carry out the RIP assay according to the product specifications. First, the HepG2 cells were collected and lysed in a full RIP lysis buffer. Cell extracts were then incubated with RIP buffer containing magnetic beads conjugated to human AGO2 antibodies (ab32381, abcam, Cambridge, United Kingdom), and IgG antibody (ab6702, abcam, Cambridge, United Kingdom) was used as controls. The samples were incubated with protease K and oscillated to digest the protein and isolate the immunoprecipitated RNA. The concentration of RNA was then measured using a NanoDrop spectrophotometer and real-time PCR analysis of the purified RNA was performed.

### Dual Luciferase Reporter Gene Assay

CDK1 and CCNB1 fragments containing miR-199a-3p binding sites were amplified by PCR and cloned into the downstream of luciferase reporter gene in pmirGLO vector, which were named CDK1-WT and CCNB1-WT. CDK1-MUT and CCNB1-MUT (mutations within the binding sites) were generated using the Quickchange XL Site-Directed Mutagenesis Kit (Stratagene) according to the manufacturer’s protocol. Mimic NC and miR-199a-3p mimic were co-transfected with CDK1-WT or CDK1-MUT and CCNB1-WT or CCNB1-MUT, respectively, into HepG2 cells. After 48 h of transfection, cells were harvested and luciferase assay was performed using the dual luciferase reporter system (Promega).

### RNA Pull-Down

RNA pull-down measurements were performed using the Pierce TM Magnetic RNA-Protein Pull-Down Kit (Millipore) according to the manufacturer’s instructions. In brief, HepG2 cells were transfected with 3′-terminal biotin-labeled LNC00346 probe and its control probe. 24 h after transfection, the cells were incubated with streptomycin-coated magnetic beads. The expressions of LNC00346 and miR-199a-3p in the binding portion were determined by qRT-PCR.

### Statistical Analysis

SPSS 21 (IBM Corp., Armonk, NY, United States) was used for statistical analysis of data between different groups. All data were expressed as Mean ±SD. The comparison between two groups was analyzed by *t-*test. *P* < 0.05 was statistically significant.

## Results

### CDK1 and CCNB1 Are Possible Targets for HCC

In order to find the genes associated with HCC development, we firstly conducted differential analysis on GES62232 dataset in GEO database to analyze the mRNAs with significantly different expressions, and 230 DEGs in HCC were obtained (Supplementary Table S1). Figure 1A showed the expressions of the first 100 DEGs. Further analysis of KEGG function enrichment of these DEGs revealed that six genes were enriched in p53 signaling pathway (Figure 1B). P53 signaling pathway was believed to be involved in cell apoptosis, cell cycle and other activities, and many studies indicated that it was involved in tumor development (Smal et al., 1989; Meng et al., 2014). Protein interaction analysis was performed on these six genes (Figure 1C) and it was found that CDK1 and other three genes were at the core position. CDK1 and CCNB1 were chosen for the follow-up studies. The expression levels of CDK1 and CCNB1 in HCC tumor samples and normal samples from TCGA database were analyzed (Figures 1D,E) and we found that CDK1 and CCNB 1 were highly expressed in HCC, which suggested that CDK1 and CCNB1 may play important regulatory roles in HCC.

**FIGURE 1:** CDK1 and CCNB1 are possible targets for HCC. **(A)** Heat map of the first 100 DEGs expression in GSE62232 dataset from GEO database; **(B)** KEGG pathway enrichment analysis of DEGs in GSE62232 dataset; **(C)** Interaction analysis of DEGs in p53 signaling pathway, orange represents high expression and blue represents low expression; **(D,E)** CDK1 and CCNB1 gene expression in HCC samples and normal samples from TCGA database, red is the tumor sample and black is the normal sample. *represents *P* < 0.05.

### CDK1/CCNB1 Regulate Cell Cycle, Apoptosis and Invasion in HCC

We first detected the expression of CDK1 and CCNB1 in human normal liver cells L-02 and HCC cell lines HepG2, Huh-7, Hep3b, and SMMC-7721 by qRT-PCR. The results exhibited that both CDK1 and CCNB1were highly expressed in HCC cells (Figure 2A) (*P* < 0.05), and then the two HCC cell lines HepG2 and Huh-7 with higher expression of CDK1 and CCNB1 were selected for subsequent experiments. WB was used to detect the protein expressions of CDK1 and CCNB1 in L-02, HepG2 and Huh-7 cell lines (Figure 2B). Compared with L-02, the protein expressions of CDK1 and CCNB1 were significantly increased in HepG2 and Huh-7 cell lines, which was consistent with the expression trend of mRNA. In order to further study the functional role of CDK1 and CCNB1 in HCC, we established CDK1 and CCNB1 silencing cell lines and the silencing efficiency was detected by qRT-PCR (Figures 2C,D). Compared with si-NC group, CDK1 and CCNB1 were effectively silenced (*P* < 0.05), and si-CDK1-2 and si-CCNB1-2 sequences with better silencing efficiency were selected for subsequent experiments. Then, FCM was performed to detect apoptosis in si-NC group, si-CDK1 group and si-CCNB1 group (Figure 2E). The results showed that silencing CDK1/CCNB1 promoted apoptosis of HepG2 and Huh-7 cells in HCC (*P* < 0.05). After studying the effect of CDK1/CCNB1 on apoptosis of HCC cells, its effects on cell invasion and cell cycle were also studied. Transwell assay was used to determine cell invasion (Figure 2F). The results exhibited that the invasion ability of HCC cells decreased significantly after CDK1/CCNB1 was silenced (*P* < 0.05). Then FCM was used to detect the cell cycle (Figure 2G). The proportion of cells in G0/G1 phase in the si-CDK1 group and si-CCNB1 group increased significantly, and the proportion of cells in S phase decreased greatly (*P* < 0.05). In conclusion, silencing CDK1 or CCNB1 can promote the apoptosis of HCC cell lines HepG2 and Huh-7, inhibit cell invasion, and block cells in G0/G1 phase.

**FIGURE 2:** Expression and regulation of CDK1 and CCNB1 in HCC cells. **(A)** The expressions of CDK1 and CCNB1 in normal human cells and four HCC cell lines were detected by qRT-PCR; **(B)** The protein expressions of CDK1 and CCNB1 in HepG2 and Huh-7 were detected by WB; **(C,D)** The silencing efficiency of CDK1 and CCNB1 was measured by qRT-PCR; Cells development in each group was detected by FCM and Transwell assays (100×). **(E)** Cell apoptosis; **(F)** Cell invasion; **(G)** Cell cycle. *means *P* < 0.05. Representative of three independent experiments.

### CDK1/CCNB1 Affect the Apoptosis, Invasion and Cell Cycle of HCC by Regulating p53 Pathway

After determining the biological function of CDK1/CCNB1 on HCC cells, we investigated the effect of CDK1 and CCNB1 on HCC cells by regulating p53 pathway. The transfected HepG2 cells with the highest CDK1 expression were divided into si-NC + DMSO group, si-NC + PFT β group, si-CDK1 + DMSO group, si-CDK1 + PFT β group, and transfected Huh-7 cells with the highest CCNB1 expression were divided into si-NC + DMSO group, si-NC + PFT β group, si-CCNB1 + DMSO group, si-CCNB1 + PFT β group. First, WB was used to detect the protein expressions of CDK1, CCNB1, p53 and p21 in cells in each group. As displayed in Figures 3A,B, silencing CDK1/CCNB1 can promote the protein expressions of p53 and p21 in cancer cells (*P* < 0.05), while the result was reverse with the addition of PFT β, a p53 pathway inhibitor. This result indicated that CDK1/CCNB1 could negatively regulate p53 signaling pathway.

**FIGURE 3:** CDK1 and CCNB1 affect the apoptosis, invasion and cell cycle of HCC by regulating p53 pathway. **(A)** The protein expressions of CDK1, p53 and p21 in HepG2 cells were detected by WB; **(B)** The protein expressions of CCNB1, p53 and p21 in Huh-7 cells were detected by WB; Cells development in each group was detected by FCM and Transwell assays (100×). **(C,D)** Cell apoptosis; **(E,F)** Cell invasion; **(G,H)** Cell cycle. *means *P* < 0.05.

In order to study the function of this regulation in HCC, we used FCM to detect the apoptosis of each group (Figures 3C,D). The results displayed that compared with the si-NC + DMSO group, the apoptosis rate of the si-NC + PFT β group was significantly reduced. CDK1 or CCNB1 silencing group can eliminate the inhibitory effect on apoptosis of pathway inhibitor group. Then Transwell was used to detect the cell invasion of each group (Figures 3E,F). The results showed that PFT β promoted invasive ability of cancer cells while CDK1 or CCNB1 silencing group canceled out the promoting effect of PFT β on invasion ability of HepG2 or Huh-7 cells (*P* < 0.05). Finally, FCM was used to detect the cell cycle (Figures 3G,H). We observed that the proportion of cells in the G0/G1 phase in the si-NC + PFT β group decreased significantly, while that in the S phase increased significantly. Silencing CDK1 or CCNB1 blocked cell cycle and eliminates the effect of PFT β. These results suggested that inhibiting CDK1/CCNB1 could promote invasion, inhibit apoptosis and regulate cell cycle of HCC cells by blocking the p53 signaling pathway.

### miR-199a-3p Targeted Inhibits Both CDK1 and CCNB1 Expression

In order to investigate the upstream miRNAs that regulate CDK1/CCNB1, the TargetScan database was further used to predict the upstream regulatory miRNAs of CDK1 and CCNB1. At the same time, a miRNA expression dataset GSE74618 of HCC was obtained through the GEO database and analyzed. Finally, two miRNAs that were significantly down-regulated in HCC were obtained. The microarray analysis results and TargetScan prediction results were intersected (Figure 4A) and it was found that there was only one miRNA that was miR-199a-3p in the intersection. The expression level of miR-199a-3p in GSE74618 dataset was significantly lower in HCC samples (Figure 4B). QRT-PCR was used to detect the expression of miR-199a-3p in human normal liver cells L-02 and HCC cell lines HepG2 and Huh-7 (Figure 4C). The result showed that miR-199a-3p was significantly lowly expressed in HCC cells (*P* < 0.05). Next, the binding sites of miR-199a-3p and CDK1 or CCNB1 were predicted by bioinformatics website, respectively, to explore the targeting relationship between mir-199a-3p and CDK1 or CCNB1 (Figure 4D). miR-199a-3p can bind to the 3′UTR of CDK1 or CCNB1, respectively. Then RIP assay was performed on HepG2 cells to detect whether miR-199a-3p could bind with CDK1 or CCNB1, as shown in Figure 4E. Compared with IgG antibodies, CDK1 and CCNB1 enriched in AGO2 antibody group were significantly increased (*P* < 0.05). Moreover, dual luciferase reporter gene assay was used to verify the targeted binding relationship (Figure 4F). Compared with the mimic NC group, the relative fluorescence activity of miR-199a-3p mimic was significantly decreased in the co-transfection group with CDK1-WT or CCNB1-WT, indicating that miR-199a-3p could target CDK1 and CCNB1, respectively. In addition, HepG2 cell line was transfected into NC mimic group and miR-199a-3p mimic group. Expressions of miR-199a-3p, CDK1 and CCNB1 were detected by qRT-PCR (Figure 4G), and protein expressions of CDK1 and CCNB1 were detected by WB (Figure 4H). Overexpression of miR-199a-3p resulted in down-regulation of mRNA and protein expression levels of CDK1 and CCNB1 (*P* < 0.05). These results proved that miR-199a-3p inhibit CCNB1 and CDK1 expressions.

**FIGURE 4:** miR-199a-3p targeted inhibited CDK1 and CCNB1 expression. **(A)** The miRNAs that regulate CDK1 and CCN1 were predicted by TargetScan and intersections with significantly down-regulated expression in GSE74618 of HCC; **(B)** miR-199a-3p expression in GSE74618 dataset, black represents the normal sample and red represents the tumor sample; **(C)** The expression of miR-199a-3p in L-02, HepG2 and Huh-7 cell lines was detected by qRT-PCR; **(D)** The binding sites of miR-199a-3p and CDK1 or CCNB1; **(E)** RIP assay was used to detect whether miR-199a-3p could bind with CDK1 and CCNB1; **(F)** Dual luciferase reporter gene assay was used to verify the targeted binding relationship between miR-199a-3p and CDK1/CCNB1; **(G)** The expressions of miR-199a-3p, CDK1 and CCNB1 in HepG2 cells were detected by qRT-PCR; **(H)** Protein expressions of CDK1 and CCNB1 in HepG2 cells was detected by WB. *represents *P* < 0.05.

### miR-199a-3p Affects the Apoptosis, Invasion and Cell Cycle of HCC Through Targeting CDK1 and CCNB1

Next, in order to explore the effect of miR-199a-3p on HCC by targeting CDK1 and CCNB1, HepG2 cells were transfected into inhibitor NC + si-NC, miR-199a-3p inhibitor + si-NC, inhibitor NC + si-CDK1, miR-199a-3p inhibitor + si-CDK1 groups, and Huh-7 cells were transfected into inhibitors NC + si-NC, miR-199a-3p inhibitor + si-NC, inhibitor NC + si- CCNB1, miR-199a-3p inhibitor + si-CCNB1 groups. QRT-PCR was used to detect the expressions of miR-199a-3p and CDK1 in HepG2 cells, as well as expressions of miR-199a-3p and CCNB1 in Huh-7 cells. As exhibited in Figures 5A,B. Silencing miR-199a-3p significantly up-regulated the expressions of CDK1 and CCNB1 (*P* < 0.05). WB was performed to examine the protein expressions of p53 and p21 in cells of each group (Figures 5C,D). The results revealed that silencing miR-199a-3p inhibited the protein expressions of p53 and p21, while simultaneously silencing CDK1/CCNB1 offset the inhibitory effect of silencing miR-199a-3p (*P* < 0.05).

**FIGURE 5:** miR-199a-3p affects the apoptosis, invasion and cell cycle of HCC through CDK1 and CCNB1. The mRNA and protein expressions of miR-199a-3p, CNK1, CCNB1, p53 and p21 in each group were detected by qRT-PCR and WB, respectively. Cells development in each group was detected by FCM and Transwell assays (100×). **(A)** MRNA expressions of miR-199a-3p and CDK1 in HepG2 cells; **(B)** MRNA expressions of miR-199a-3p and CCNB1 in Huh-7 cells; **(C)** The protein expressions of p53 and p21 in HepG2 cells; **(D)** The protein expressions of p53 and p21 in Huh-7 cells; **(E,F)** Cell apoptosis; **(G,H)** Cell invasion; **(I,J)** Cell cycle. *represents *P* < 0.05. Representative of three independent experiments.

Functionally, FCM was used to detect the apoptosis rate (Figures 5E,F), compared with the inhibitor NC + si-NC group, the miR-199a-3p inhibitor + si-NC group had a significantly lower apoptosis rate, while inhibitor NC + si-CDK1 and the inhibitor NC + si-CCNB1 group had a significantly increased apoptosis rate. The co-transfection groups of miR-199a-3p inhibitor with si-CDK1 or si-CCNB1 offset the effect of both on apoptosis. Similarly, Transwell was used to measure cell invasion (Figures 5G,H). The results showed that silencing miR-199-3p could promote the invasion of HCC cells while silencing CDK1/CCNB1 would counteract the promoting effect of miR-199-3p (*P* < 0.05). Finally, FCM was used to detect the cell cycle (Figures 5I,J). We found that the cell ratio in G0/G1 phase in the miR-199a-3p inhibitor group was significantly reduced, and the cell ratio in S phase was significantly increased. While silencing CDK1 or CCNB1 improved miR-199a-3p inhibitory effect on cell cycle arrest.

In conclusion, miR-199a-3p activated the p53 signaling pathway by targeted inhibiting the expressions of CDK1 and CCNB1, thus promoting the apoptosis of HepG2 or Huh-7 cells, inhibiting the invasion and regulating cell cycle.

### LINC00346 Regulates the Expression of CDK1 and CCNB1 by Sponging miR-199a-3p

After confirming that miR-199a-3p regulated HCC cells by targeting CDK1/CCNB1, we then used the RNA22 database to find the corresponding lncRNA to miR-199a-3p and found that it was regulated by LINC00346. Moreover, studies have reported that LINC00346 was significantly negatively correlated with the survival of HCC patients, and could play a regulatory role through the mechanism of ceRNA (Zhang et al., 2015). These results suggested that LINC00346 may target and regulate the expression of CDK1 and CCNB1 by sponging miR-199a-3p, thereby affecting the p53 signaling pathway and ultimately participating in the development of HCC. For verification, the binding sites of LINC00346 and miR-199a-3p (Figure 6A) were predicted by bioinformatics website, and RNA pull-down assay was performed to verify the interaction between LINC00346 and miR-199a-3p in HepG2 cells. As shown in Figure 6B, both LINC00346 and miR-199a-3p were significantly enriched in the biotin-labeled LINC00346 drop-down conjugate (*P* < 0.05), indicating that LINC00346 could directly bind to miR-199a-3p. Then RIP was conducted to detect the binding of LINC00346 and miR-199a-3p. As displayed in Figure 6C, compared with IgG antibody, LINC00346 and miR-199a-3p enriched in AGO2 antibody group were significantly increased (*P* < 0.05). After silencing LINC00346, the relative enrichment of LINC00346 was significantly decreased, while that of CDK1 and CCNB1 was significantly increased (Figure 6D).

**FIGURE 6:** LINC00346 regulates the expression of CDK1 and CCNB1 by sponging miR-199a-3p. **(A)** The binding sites of LINC00346 and miR-199a-3p; **(B)** RNA pull-down assay was used to verify the interaction between LINC00346 and miR-199a-3p, red letters indicate predicted binding sites of LINC00346 and mRNA-199a-3p **(C)** RIP was used to detect the binding of LINC00346 and miR-199a-3p in each group; **(D)** RIP was used to detect changes in LINC00346, CDK1 and CCNB1 binding to miR-199a-3p in each group; **(E)** Expression changes of LINC00346, miR-199a-3p, CDK1 and CCNB1 after LINC00346 silencing were detected by qRT-PCR; **(F)** The expressions of LINC00346, miR-199A-3p, CDK1 and CCNB1F in each group were detected by qRT-PCR and WB, respectively: The expressions of LINC00346, miR-199a-3p, CDK1 and CCNB1; **(G)** Protein expressions of CDK1 and CCNB1. *represents *P* < 0.05.

We then determined whether LINC00346 could modulate the expression of miR-199a-3p in HCC cells. HepG2 cells were transfected into si-NC and si-LINC00346 groups. QRT-PCR was used to detect the changes of LINC00346, miR-199a-3p, CDK1 and CCNB1 after silencing LINC00346. As shown in Figure 6E, silencing LINC00346 promoted the expression of miR-199a-3p and decreased the expression of CDK1 and CCNB1 (*P* < 0.05). Finally, HepG2 cells were transfected into si-NC + inhibitor NC, si-LINC00346 + inhibitor NC, si-NC + miR-199a-3p inhibitor, si-LINC00346 + miR-199a-3p inhibitor groups and the expressions of LINC00346, miR-199a-3p, CDK1, and CCNB1 in each group were detected (Figure 6F). WB was used to detect the protein expressions of CDK1 and CCNB1 in each group (Figure 6G). The results revealed that the mRNA and protein expressions of CDK1 and CCNB1 were significantly down-regulated after silencing LINC00346, and those were significantly up-regulated after silencing miR-199a-3p. Silencing LINC00346 and miR-199a-3p simultaneously canceled out the effects of silencing CDK1 and CCNB1 expression (*P* < 0.05). In conclusion, LINC00346 promoted the expression of CDK1 and CCNB1 by sponging miR-199a-3p.

### LINC00346 Affects the Apoptosis, Invasion and Cell Cycle of HCC by Regulating the Expression of CDK1 and CCNB1

Finally, we explored the effect of LINC00346 on CDK1 and CCNB1 regulation on HCC. HepG2 cells were transfected and divided into si-NC group and si-LINC00346 group. Protein expressions of p53 and p21 were detected by WB (Figure 7A). The results showed that silencing LINC00346 promoted the protein expressions of p53 and p21 (*P* < 0.05). Functionally, the apoptotic rate was detected by FCM (Figure 7B) and observed that the apoptosis rate in si-LINC00346 group was significantly increased (*P* < 0.05). Cell invasion was detected by Transwell (Figure 7C). The results exhibited that silencing LINC00346 decreased the invasion ability of HCC cells (*P* < 0.05). FCM was used to detect the cell cycle (Figure 7D), we found that the cell proportion of G0/G1 phases in the si-LINC00346 group increased significantly, and the cell proportion of S phase decreased significantly. The results showed that silencing LINC00346 promoted p53 signaling pathway, promoted apoptosis, inhibited invasion, and blocked cells in G0/G1 phase.

**FIGURE 7:** Silencing LINC00346 affects the apoptosis, invasion and cell cycle of HCC. **(A)** Protein expressions of p53 and p21 in each group were detected by WB; Cells development in each group was detected by FCM and Transwell assays (100×). **(B)** Cell apoptosis; **(C)** Cell invasion; **(D)** Cell cycle. *represents *P* < 0.05.

HepG2 cells after transfection were then grouped into oe-NC + si-NC, oe-LINC00346 + si-NC, oe-LINC00346 + si-CDK1, and oe-LINC00346 + si-CCNB1. The expressions of LINC00346, CDK1 and CCNB1 in each group were detected by qRT-PCR (Figure 8A). The results indicated that the expressions of LINC00346, CDK1 and CCNB1 in the oe-LINC00346 + si-NC group were significantly up-regulated compared with those in the oe-NC + si-NC group (*P* < 0.05). Compared with oe-LINC00346 + si-NC group, the expression of CDK1 in oe-LINC00346 + si-CDK1 group and CCNB1 in oe-LINC00346 + si-CCNB1 group were significantly down-regulated (*P* < 0.05). WB was performed to detect the protein expressions of CDK1, CCNB1, p53 and p21 in each group (Figure 8B). The results revealed that overexpression of LINC00346 promoted the expressions of CDK1 and CCNB1 and inhibited the expressions of p53 and p21 (*P* < 0.05). FCM was also used to detect the apoptosis rate (Figure 8C). Overexpression of LINC00346 inhibited cell apoptosis, while silencing CDK1 and CCNB1 reversed the inhibitory effect of LINC00346 overexpression on apoptosis. Transwell was conducted to detect cell invasion (Figure 8D). Overexpression of LINC00346 promoted cell invasion, while the co-transfection group of over-expressing LINC00346 and silenced CDK1 or CCNB1 reversed the promotion effect of over-expressing LINC00346. FCM was used to measure cell cycle (Figure 8E). We found that compared with the oe-NC + si-NC group, the cell ratio of G0/G1 phase in the oe-LINC00346 group was significantly reduced while the cell ratio in S phase was significantly increased, and silencing CDK1 or CCNB1 improved the inhibitory effect of overexpression of LINC00346 on cell cycle arrest. The results above showed that overexpression of LINC00346 promoted the expressions of LINC00346, CDK1, and CCNB1 and invasion, inhibited the p53 pathway and apoptosis, and blocked cells in the S phase. These results indicated that LINC00346 could block the p53 signaling pathway by promoting the expressions of CDK1/CCNB1, thereby promoting the invasion of cancer cells, inhibiting apoptosis and regulating cell cycle.

**FIGURE 8:** LINC00346 affects the apoptosis, invasion and cell cycle of HCC by regulating the expression of CDK1 and CCNB1. The mRNA and protein expressions of LINC00346, CNK1, CCNB1, p53 and p21 in each group were detected by qRT-PCR and WB, respectively. Cells development in each group was detected by FCM and Transwell assays (100×). **(A)** The expressions of LINC00346, CDK1 and CCNB1; **(B)** Protein expressions of CDK1, CCNB1, p53 and p21; **(C)** Cell apoptosis; **(D)** Cell invasion; **(E)** Cell cycle. *represents *P* < 0.05.

## Discussion

Because of the high recurrence and metastasis rates, the overall survival of HCC patients remains low, and the study of molecular therapies for HCC has been a hot topic (Setshedi et al., 2018). This study demonstrated that CDK1 and CCNB1 were highly expressed in HCC tissues and cells through bioinformatics analysis combined with cell experiments, which was consistent with previous results (Wu et al., 2018; Gu et al., 2019). Then, we analyzed the effects of CDK1 and CCNB1 on the biological behavior of HCC, and found that CDK1 and CCNB1, as two oncogenes, could inhibit the apoptosis of HCC cells and promote cell invasion. These two genes also play a carcinogenic role in other cancers. Yang et al. put forward that the expression of CDK1 as an oncogene would increase with the progressive deterioration of epithelial ovarian cancer (Yang et al., 2016). Ding et al. (2014) demonstrated that CCNB1 can act as a biomarker of ER + breast cancer and play an oncogenic role in the occurrence of ER + breast cancer (Ding et al., 2014). These results indicated that CDK1/CCNB1 played an important role as an oncogene in a variety of cancers including HCC.

In exploring the specific molecular mechanism of CDK1/CCNB1 in regulating cancer, Zhang et al. revealed that CCNB1 could affect the cell cycle and apoptosis of pancreatic cancer cells by regulating p53 signaling pathway (Zhang H. et al., 2018). Qin G et al. reported that the p53 signaling pathway may be regulated by multiple genes to affect the development of liver cells (Qin et al., 2019). In addition, KEGG pathway enrichment analysis (Figure 1B) showed that multiple DEGs, including CDK1/CCNB1, were enriched in the p53 signaling pathway. Therefore, we speculated that CNK1/CCNB1 might regulate the occurrence of HCC by affecting p53 signaling pathway. We had conducted several experiments to verify this hypothesis, and the results showed that silencing CDK1/CCNB1 could promote the protein expressions of p53 and p21, thus promoting the apoptosis and inhibiting the invasion of HCC cells. These results all suggested that CDK1 and CCNB1 affected the apoptosis, invasion and cell cycle of HCC by regulating p53 signaling pathway.

In order to further explore the genes related to CDK1/CCNB1, we proved the signal axis of LINC00346-miR-199a-3p-CDK1/CCNB1 through bioinformatics analysis and molecular experiments and found that miR-199a-3p could bind to the 3′UTR of CDK1 and CCNB1. Meanwhile, the targeted relationship was verified by the dual luciferase reporter gene assay, and the results of WB confirmed that miR-199a-3p inhibited the expressions of CDK1 and CCNB1. The results are consistent with the results of previous studies. Ma et al. (2019) reported that miR-199a-3p is poorly expressed in HCC cells and HEIH silence suppressed the activation of mTOR signaling via upregulating miR-199a-3p (Ma et al., 2019). Ren et al. (2016) reported that miR-199a-3p could inhibit the proliferation of HCC cells by targeted down-regulating YAP1 expression (Ren et al., 2016). Our study on the regulatory effect of miR-199a-3p on HCC also found that miR-199a-3p could activate the p53 signaling pathway by targeting the expressions of CDK1/CCNB1, thereby inhibiting the development of HCC.

In the study of LINC00346 on HCC, we found that LINC00346 significantly promoted the invasion and inhibited cell apoptosis of HCC through the competitive adsorption of miR-199a-3p to promote the expressions of CDK1/CCNB1. In recent years, lncRNAs analysis and functional assays for various types of cancer have provided increasing evidence supporting the critical role of lncRNAs in HCC tumor growth and progression, such as HOTAIR (Hu et al., 2018), MALAT1 (Tao et al., 2018) and TUG1 (Sun et al., 2018). Previous studies have found that LINC00346 is up-regulated in HCC tissues (Zhang et al., 2015). As a gene regulator, lncRNA regulates gene expression through a variety of mechanisms, one of which is sponging miRNA to up-regulate or down-regulate miRNA expression. Previous studies have reported that the LINC00346-miR-10a-5p-CDK1 axis may be an important mechanism for HBV-related HCC, and genes in this ceRNA axis may be potential prognostic biomarkers and therapeutic targets (Li et al., 2019). The effects of the ceRNA axis of LINC00346-miR-199a-3p-CDK1/CCNB1 on cell invasion, apoptosis and cell cycle of HCC was demonstrated in this study, which further proved the role of LINC00346 as an oncogene in HCC, and the mechanism of HCC was further investigated.

## Conclusion

In conclusion, LINC00346 has a positive regulatory effect on HCC. LINC00346 can regulate CDK1/CCNB1 to inhibit apoptosis, promote cell invasion and regulate cell cycle of HCC by targeting miR-199a-3p, while LINC00346-miR-199a-3p-CDK1/CCNB1 signal axis can regulate p53 signaling pathway. This result provides a deeper understanding of LINC00346’s role in HCC, and lays the foundation for searching new targeted therapies for HCC.

## Data Availability Statement

The data used to support the findings of this study are included within the article. The data and materials in the current study are available from the corresponding author on reasonable request.

## Author Contributions

JJ contributed to the study design. HX conducted the literature search. WL and XX wrote the article. HL and FW revised the article.

## Conflict of Interest

The authors declare that the research was conducted in the absence of any commercial or financial relationships that could be construed as a potential conflict of interest.

## Footnotes

1 https://www.ncbi.nlm.nih.gov/geoprofiles/

2 https://string-db.org

3 https://www.cancer.gov/

4 http://gepia.cancer-pku.cn/

5 http://www.targetscan.org/vert_71/

6 http://www.rna-society.org/raid2/index.html

7 https://cm.jefferson.edu/rna22/

## Supplementary Material

TABLE S1 230 differential genes screened by differential analysis of GES62232 dataset in GEO database.
